The article "Clinical Features of Acute Coronary Syndrome in Patients with Coronary Heart Disease and Its Correlation with Tumour Necrosis Factor in Cardiology" was published in 2022. Journal: Comput Math Methods Med.

# Clinical Features of Acute Coronary Syndrome in Patients with Coronary Heart Disease and Its Correlation with Tumour Necrosis Factor in Cardiology

**DOI:** 10.1155/2022/3439768

**Published:** 2022-06-30

**Authors:** Run Guo, Tingting Wu, Nan Zheng, Yanfang Wan, Jun Wang

**Affiliations:** Department of Cardiovascular Medicine, Cangzhou Central Hospital, Cangzhou, 061000 Hebei, China

## Abstract

Tumour necrosis factor (TNF) levels are higher in patients who have experienced an acute ischemic stroke. Greater levels of TNF may not be linked to an increased risk of recurrent coronary events in the stable phase after myocardial ischemia (MI). Coronary atheroma is connected to endothelial and smooth muscle cells, as well as macrophages that emit the multifunctional cytokine tumour necrosis factor (TNF). Transplanted tumours become more vulnerable when TNF-*α* was first recognized to have a function in hemorrhagic necrosis. TNF-*α* has been demonstrated to induce heart failure, pulmonary edoema, and cardiomyopathy in people with advanced heart failure when it is elevated in the bloodstream. It has been postulated that prolonged overexpression of TNF-*α* after ischemia may contribute to poor cardiac outcomes by increasing TNF-*α* when the myocardium undergoes both temporary ischemia and reperfusion. A rise in TNF levels has been seen after a myocardial infarction, but it is unclear if these higher levels, found months after the initial event, are associated with an increased risk of subsequent heart attacks. We looked at TNF levels in the blood of 270 patients with coronary heart disease in the Chinese Hypertension League's Cholesterol and Recurrent Events (CARE) experiment to see if this notion held true. Recurrent coronary syndrome and coronary mortality were monitored prospectively in the participants. The min max imbalance normalization can be used to assess a patient's baseline characteristics, including hormone and cholesterol test results. Type 2 stimulant connection to aggregate the TNF-signaling qualities and fuzzy techniques was applied. There may now be enough preliminary evidence from the crucial bundle neural network analysis to identify the risk of coronary heart disease associated with TNF pregeneration studies. The tests were assessed using a variety of methods and performance metrics in a Matlab environment.

## 1. Introduction

In addition to hypertension, dyslipidemia, diabetes, ischemic heart disease, postpartum cardiomyopathy, and congenital defects, a number of variables contribute to the onset of acute coronary syndrome. Heart tissue injury may be refurbished by activating the heart's innate immune system. Innate immunity is activated following heart damage, as shown by an increase in the repertory of proinflammatory cytokines. Heart stress is associated with the production of proinflammatory cytokines, such as TNF-*α*, TGF-*β*, and the interleukin (IL) family, which includes IL-1, 12, 8, and 18. Proinflammatory cytokines, which have been demonstrated to have beneficial effects on tissue repair, play a role in cardiac remodeling. An injury's anti-inflammatory response occurs after the initial proinflammatory stage, which is becoming more obvious. Localized smooth muscle injury and increased leukocyte extravasation prolong the proinflammatory cycle because of the diverse and unique nature of cardiac stress, which increases the proinflammatory response. Chronic inflammation, which is aggravated by diseases like hypertension, diabetes, and other comorbidities, may result if the proinflammatory process is allowed to continue unchecked. A supply of proinflammatory cytokines must be established in heart tissue by macrophages in order to sustain chronic inflammation. Excessive production and discharge into the circulation of cytokines put other organs at danger. TNF-*α* and IL-6 have been suggested as potential markers of heart failure in a number of studies. Furthermore, endothelial and smooth muscle cells, as well as macrophages, generate tumour necrosis factor- (TNF-*α*), a multifunctional circulating cytokine, which is associated with coronary atherosclerosis. When TNF-*α* was originally recognized to have a role in hemorrhagic necrosis, transplanted tumours were shown to be more vulnerable. TNF-*α*, for instance, is elevated in severe heart failure and may induce pulmonary edoema, left ventricular dysfunction, and cardiomyopathy in experimental settings. TNF-*α* overexpression during ischemia has been hypothesized to contribute to poor cardiac outcomes. Both transient cardiac ischemia and reperfusion cause an increase in TNF-*α* level in the myocardium. However, it is not known whether higher TNF-*α* levels discovered months after a MI are connected to an increased risk of recurrent coronary events. This has been seen in several studies. This hypothesis was tested by including patients with increased levels of TNF-*α* in the Cholesterol and Recurrent Events (CARE) experiment. The goal of this study was to identify recurrences of MI and cardiac death in patients with acute coronary syndromes. To identify patients who had recurrent coronary episodes and those who did not, we examined post-MI TNF-*α* level in nested case-control analysis using the paramount bundle neural network (PBNN).

The article "Clinical Features of Acute Coronary Syndrome in Patients with Coronary Heart Disease and Its Correlation with Tumour Necrosis Factor in Cardiology" was published in 2022. Journal: Comput Math Methods Med.

The paper's arrangement is as follows: Related work is summarized briefly in Section 2. Problem statement is described in Section 3. The implemented methods for performance analysis are presented in Section 4.  Section 5 concludes the paper.

## 2. Related Works

More research on TNF production and its link to cardiovascular disease has been published by other authors. The author of [1] looked into these abnormalities in metabolism and fibrinolysis to see if TNF was involved. TNF levels were measured in 45-year-old male postinfarction patients and matched population-based controls. Patients had greater TNF plasma levels (4.1-4.6) than healthy controls (2.5-0.4 pg/mL). People with hyperlipidemia were shown to have higher levels of TNF-*α*, which was associated to higher levels of VLDL triglyceride and HDL cholesterol. This medication lowered VLDL triglyceride levels and elevated HDL cholesterol, but it had no impact on TNF-*α* concentrations. TNF concentrations were connected to glucose and proinsulin levels before and after glucose ingestion, as well as glucose and proinsulin levels after glucose consumption. In [2], this study employed CTRP 9 as well as pentraxin 3 (PTX3) to examine the diagnostic and prognostic value of C1q/tumour necrosis factor-related protein 9 in patients with acute coronary syndromes (ACS). A total of 137 people were found to have heart disease or chest pain. We divided those with ACS into one group and those with noncardiac chest pain (NCCP) into another group as “controls.” An ELISA test was performed to check the blood levels of CTRP9 and PTX3 to see how they compare to other ACS-related indices and whether or not they may be utilized to diagnose ACS and predict a poor prognosis. In [3], lncRNA MALAT1 and miR-125b were examined in connection to coronary heart disease risk, severity, and prognosis in order to assess the association between these two genes (CHD). In [4], among individuals from the Saudi population, the author found a link between serum tumour necrosis factor- (TNF-) alpha and metabolic syndrome (MetS) components. In [5], the author examined the expression of lncRNA-FA2H-2 and its association with inflammatory markers in individuals with coronary heart disease (CHD). In [6], TNF-*α* expression in SCAD was investigated using metabolic, inflammatory, and microRNA (miRNA) markers. Researchers enlisted patients with SCAD, who were then tested for their metabolic and inflammatory profiles. To determine the presence of TNF, an enzyme-linked immunosorbent assay was performed. The relative levels of expression of MiRNAs associated with inflammation and/or atherosclerosis were assessed. In [7], a biomarker for distinguishing ACS-related chest pain from non-ACS-related chest pain may be plasma sTREM-1, according to the author. To see whether plasma sTREM-1 levels might be used to predict 30-day and six-month cardiovascular outcomes in patients with early-stage ACS, the researchers set out to do this study. In [8], swine farm workers who smoke may be affected by TNF gene polymorphisms, the study's author claims. Researchers in Saskatchewan polled more than 400 full-time swine farm workers and 411 nonfarming rural inhabitants. As part of the trial, researchers collected information about participants' demographics and lifestyle, as well as lung function and blood samples. Several linear regressions were used in the statistical analysis. Polymorphisms in the promoter of the TNF gene were investigated for three different variations. In [9], patients with acute myocardial infarction (AMI) who has periodontitis and systemic inflammation are examined by the author for their relationship to a variety of indications of heart disease. In [10], molecular targets for heart disease and the molecular mechanisms that underpin it are the focus of this research. The GSE66360, GSE19339, and GSE97320 array datasets were obtained from individuals with CAD. Gene expression profiles were generated and important modules associated with coronary heart disease were revealed by weighted gene coexpression network analysis using normalizing and decreasing inconsistencies between the three datasets (WGCNA). DAVID's database for annotating, visualizing, and integrating discovery (GO) functional and KEGG pathway enrichment studies was used to identify statistically significant genetic clusters. In [11], the author's purpose was to employ intravascular ultrasound (IVUS) images and deep learning convolutional neural networks to analyze the risk factors for adverse cardiovascular events (ACVEs) in elderly patients with coronary heart disease (CHD) following percutaneous coronary intervention (PCI) (CNNs). In [12], psoriasis patients on TNFi therapy may be at decreased risk of suffering a significant adverse cardiovascular event, according to the author's research (MACE). In their retrospective cohort study using the KPSC health plan, they found at least three ICD-9 psoriasis diagnoses but no preceding MACE codes. In the study population, multivariable Cox regression was utilized to investigate the hazard ratios (HR) of MACE associated with TNFi use. In [13], meta-analysis was undertaken by the author to examine the risk of MACEs in adult plaque psoriasis patients who are exposed to biologic therapies. In [14], the author assessed the prognostic importance of EAT volume and attenuation values derived from noncontrast cardiac computed tomography. In [15], in this study, the CT plaque characteristics of ACS patients were analyzed to identify possible culprit lesions (CLs) [16]. The level of platelet activation and inflammatory reaction in coronary artery lesions in acute coronary syndrome could be predicted by serum PDGF contents in peripheral blood as well as coronary arteries, according to research findings. In patients with acute myocardial infarction, coronary sinus Ang-1 amounts may represent the seriousness of lesions. PDGF as well as Ang-1 could be designed to estimate the degree and prognosis of acute coronary syndrome patients [17]. Via many points of system interaction for miRNA control, circRNAs were implicated in the formation and progression of ACS. They believe that circRNAs could be used as a therapeutic avenue for a pathophysiological process of ACS, and that they could possibly be used as diagnosis and therapy biomarkers. They shall conduct in vitro and in vivo experiments in the long term to confirm the role of circRNAs throughout the atherosclerotic process of ACS [18]. In China, the most common way for treating CHD would be to accurately diagnose the condition utilizing contemporary medicine to assess syndrome distinction and then combining that with TCM. circRNAs as well as miRNAs were involved in the control of AS genesis and growth in various studies. CircRNA and miRNA are essential regulators of vascular function and structure, including in the development of CHD and AS [19]. Recurrent CV incidents, DR, and DN have all been highly linked with the duration of T2DM in a group with current ACS and T2DM. The existence from either DR or DN has been implicated as the cause of recurring CV incidents. Because the length of T2DM, although maintained a strong independent indicator of recurrent CV incidents, was adjusted out of the equation, the link with DR and/or DN and all these incidents were unlikely to be causal [20]. In ACS, there may be a great desire for a consistent, available, noninvasive, and hematological prognostic marker that may detect individuals with high cardiovascular disease risk and adapt treatment to particular requirements in prevention [21]. The chances of having UGIB paired with ACS were higher throughout the corresponding time while hospitalized, according to this report. Raised fibrinogen and RDW, in association with fundamental heart attacks, syncope, a large reduction in haemoglobin, and high total bilirubin levels, may alert individuals to the possibility of ACS. Individuals with UGIB can then use the Rockall rating and the Glasgow Blatchford rating to forecast the danger of UGIB paired with ACS in a timely way.

The article "Clinical Features of Acute Coronary Syndrome in Patients with Coronary Heart Disease and Its Correlation with Tumour Necrosis Factor in Cardiology" was published in 2022. Journal: Comput Math Methods Med.

## 3. Problem Statement

Congestive heart failure is associated with an increased production of proinflammatory cytokines. TNF is an important proinflammatory cytokine that causes heart failure by suppressing the body's natural anti-inflammatory responses and disrupting the homeostatic system. In this review, we lay forth the current understanding of how TNF causes heart failure. TNF and IL-6 biomarkers have been connected to the severity of heart failure, suggesting that they could be employed as biomarkers in the future. The mechanisms by which TNF leads to cardiac dysfunction and failure have been the subject of recent research. However, the algorithm's participation in the current technique was little, and it will take longer to complete the procedure. Thus, an effective technique is needed to address all of the current research gaps.

### 3.1. Proposed Methodology

To better understand the relationship between TNF and heart failure, researchers have examined the cytokine's potential therapeutic uses and as a biomarker for the disease. TNF-*α* signalling in cells is mediated in part by NF-B, highlighting the dual function of TNF-*α* in cardiac physiology and disease once again. Two cognate receptors, TNF receptor 1 or 2, mediate TNF's biological actions farther down the line (TNFR1 or 2). TNF-induced TNFR1 activation is supposed to be harmful, whereas TNFR2-induced activation is thought to be beneficial, and the relative ratio of their expression in a given tissue system may alter phenotypes.

The TNF production process is depicted in Figure 1. It is also known that various cells can shed soluble TNFR1 or TNFR2 to produce TNFR1 or TNFR2 signalling molecules (sTNFRs). As a result, the pool of TNF accessible for binding and activating cell membrane TNFRs may be depleted. The importance of these sTNFRs in overall cardiac pathophysiology, however, has yet to be determined. TNF-*α* is an inflammatory ligand that comes in two forms: membrane-bound and secreted. This further complicates pathophysiology development. Even while TNF signalling is complicated, several studies have demonstrated that cardiomyocyte-specific production of TNF causes in reduced cardiac function that is dose dependent on the genetic. It will be mentioned later in the review how studies have consistently established that TNF-*α* exerts unfavourable inotrope effects in vitro and in vivo. Evidence like this suggests that TNF's proinflammatory effects on the beta-adrenergic receptor (AR) system may be the cause of the adverse inotropic phenotype associated with acute coronary syndrome. The overall representation of the suggested framework is illustrated in Figure 2.

#### 3.1.1. Dataset

The CARE trial, which assessed the efficiency of 40 mg of pravastatin daily in the secondary prevention of cardiovascular disease, was utilized by the researchers for this investigation, which included 4159 persons who previously had a MI. Double-blind placebo control was used in the experiment's design. Ejection fraction of at least 25% and absence of clinical signs of congestive heart failure made post-MI patients between the ages of 21 and 75 years eligible for CARE if the qualifying index event occurred between 3 and 20 months before randomization. In this investigation, death from cardiovascular disease was the primary metric of interest. It was required that participants in the CARE study have an LDL cholesterol level between 115 and 175 mg/dL to be eligible for randomization. Prerandomization visits were used to collect blood samples. For the duration of the testing process, samples were stored at 80°C. Prior to randomization, the cytokine TNF-*α* was examined in CARE study participants with recurrent MI or death from coronary heart disease during a 5-year follow-up period (cases) and 272 age- and sex-matched study participants who had no recurrent coronary events throughout the prerandomization period (controls). Each case and control person's frozen plasma was tested for TNF using commercially available quantitative enzyme immunoassays. TNF concentrations as low as 0.1 pg/mL have been detected, with a coefficient of variance ranging from 5% to 8%. Blood samples were evaluated in pairs in order to reduce inter-assay variability and eliminate systematic bias. The lab staff had no idea whether the samples were from a case or a control group. TNF-*α*, total lipid, blood pressure, and future TNF-*α* production variations between case and control individuals were assessed using the critical bundle neural network. Based on their medical histories, the patients were divided into two groups: A (136) and B (64). A greater number of abnormal coronary events or symptoms were seen in group A, whereas a greater number of abnormal coronary events or symptoms were observed in group B. The patient characteristics are represented in Table 1.

The article "Clinical Features of Acute Coronary Syndrome in Patients with Coronary Heart Disease and Its Correlation with Tumour Necrosis Factor in Cardiology" was published in 2022. Journal: Comput Math Methods Med.

#### 3.1.2. Preprocessing

Sizing distance and error analysis are two primary preprocessing theories that are used to establish relationships that allow accurate predictions to be made from data collected on processes or models, as well as to determine the type of relationship between each piece of information in order to collect the most relevant data for analysis. The data dimensions in which each relevant quantity involved in phenomena is represented provide the basis for error analysis. Because of this, one of the primary purposes of employing min max imbalance normalization is to produce an ordered errorless result from dimensionless words that can be analyzed. It was necessary to first set up the dimensionless variables in this example by,

(1) $$\begin{array}{c} \text{Ord}≔O\left(A\left(Q\right)=+\left|Q\left(T\right)=w\right.\right)-O\left(A\left(Q\right)=+\left|Q\left(T\right)=b\right.\right), \end{array}$$

where *A* = order function, *q* is the iterative error, *w* is the data variation, *T* is the dimensionless terms, and *b* is the backorder error.

Equation (1) can be re-arranged as follows,

(2) $$\begin{array}{c} \text{ord}\left(D\right)≔\frac{\left|\left\{Q\in D\left|Q\left(T\right)=w,Q\left(\text{Class}\right)=+\right.\right\}\right|}{\left|Q\in D\left|Q\left(T\right)=w\right.\right|}-\frac{\left|Q\in D\left|Q\left(T\right)=b,Q\left(\text{Class}\right)=+\right.\right|}{\left|Q\in D\left|Q\left(T\right)=b\right.\right|}. \end{array}$$

Once the similitude distance between the two sets of data has been determined, the similarity between them may be calculated,

(3) $$\begin{array}{c} \text{dis}\left(a_{T=b}\right)\left(A,D\right)≔\frac{\left|Q\in D\left|Q\left(T\right)=w,A\left(Q\right)=+\right.\right|}{\left|Q\in D\left|Q\left(T\right)=w\right.\right|}-\frac{\left|Q\in D\left|Q\left(T\right)=b,A\left(Q\right)=+\right.\right|}{\left|Q\in D\left|Q\left(T\right)=b\right.\right|}. \end{array}$$

To arrange the equation in a proper format, there is a need to calculate the hat matrix,

(4) $$\begin{array}{c} \frac{{\bar{q}}_{1}-\bar{q_{2}}}{\sqrt{\left(t_{1}^{2}/n_{1}\right)+\left(t_{2}^{2}/n_{2}\right)}}=\frac{\text{dis}A_{\text{hat}=g}}{\sqrt{\left(t_{1}^{2}/n_{1}\right)+\left(t_{2}^{2}/n_{2}\right)}}*\frac{{\bar{q}}_{1}-\bar{q_{2}}-d_{0}}{\sqrt{\left(t_{1}^{2}/n_{1}\right)+\left(t_{2}^{2}/n_{2}\right)}}, \end{array}$$

where

(5) $$\begin{array}{c} {\bar{q}}_{1}≔\left\{Q\in D\left|Q\left(T\right)=b\right.\right\},\\ {\bar{q}}_{2}≔\left\{Q\in D\left|Q\left(T\right)=w\right.\right\}. \end{array}$$

Finally, the ordered equation was in the form of,

(6) $$\begin{array}{c} \text{acc}\left(A^{\text{Perf}}\right)-\text{acc}\left(A\right)=\frac{\min\left(d_{b},d_{w}\right)}{d}2\frac{d_{b}}{d}\frac{d_{w}}{d}\left(\text{disc}\left(A^{\text{Perf}}\right)-\text{disc}\left(A\right)\right), \end{array}$$

where

(7) $$\begin{array}{c} \text{acc}\left(A\right)=\frac{t_{o}+t_{n}}{d}=\frac{{\text{to}}_{b}+{tn}_{b}+{\text{to}}_{w}+{tn}_{w}}{d},\\ \text{dist}\left(A\right)=\frac{{\text{to}}_{w}+{go}_{w}}{d_{w}}-\frac{{\text{to}}_{b}+{go}_{b}}{d_{o}}. \end{array}$$

### 3.2. Feature Grouping

Let us assume that *A* is a discrete random variable that can take one of *b*1 ⋯ *bn* values from the set of classes. In this example, assume that *W* is a random variable that spans throughout the set of words *W* = *W*1 ⋯ *Wn*. It is possible to estimate the joint distribution *p*(*j*, *W*) using the training dataset. There are *k* clusters *W* 1, ⋯, *Wn* of TNF signalling characteristics data. We employed stimulation type 2 links fuzzy to reduce the number of signals and the size of the model. *W* should be given a random range of values.

(8) $$\begin{array}{c} \overset{⟶}{\;A}=\overset{⟶}{c}.\overset{⟶}{P^{*}}\left(j\right)-\overset{⟶}{P}\left(j\right),\\ \overset{⟶}{P}\left(j+1\right)=\overset{⟶}{P^{*}}\left(j\right)-\overset{⟶}{a}\overset{⟶}{.E}. \end{array}$$

We employ a fuzzy measure approach to match the characteristics of clusters. Although it is ideal to conserve all mutual information when building clusters of signalling features, this is impossible since a clustering inevitably reduces mutual information. If the amount of data clusters is known, then we should try to identify a grouping that reduces signalling information as little as possible.

(9) $$\begin{array}{c} \overset{⟶}{\;P}=2.\overset{⟶}{r_{1}},\\ \overset{⟶}{A}=2\overset{⟶}{d}.\overset{⟶}{r_{2}}-\overset{⟶}{d}. \end{array}$$

Our algorithm explicitly minimizes the objective function,

(10) $$\begin{array}{c} \left\{\begin{array}{c} \frac{{\text{to}}_{b}+\left(n_{b}-{go}_{b}\right)+{\text{to}}_{w}+\left(n_{w}-{go}_{w}\right)}{d}=\text{dist}\left(A\right)\\ 0\leq {\text{to}}_{b}\leq o_{b}\\ 0\leq {\text{to}}_{b}\leq n_{b}\\ 0\leq {\text{to}}_{w}\leq o_{w}\\ 0\leq {\text{to}}_{w}\leq n_{w} \end{array}.\right. \end{array}$$

There are two kinds of distances that must be calculated for each candidate: minimum and maximum. For any pair of clusters, the inter-cluster distance between them may be determined.

(11) $$\begin{array}{c} \text{Cluster}=kA=2^{\left\lfloor \log_{2}{\left(\frac{\text{dist}\left(A\right)}{a^{m}}\right)}^{1/c}\right\rfloor }. \end{array}$$

Features that may be included include pruning with a minimum distance larger than feature distance,

(12) $$\begin{array}{c} c=\underset{k}{\min}\left[\sigma \left(\frac{\text{dis}}{m\times k^{c}}\right)\right]. \end{array}$$

If any data prototype may possibly be closer to a given subspace than any other data prototype, the above technique ensures that no feature is trimmed.

(13) cUs=C.RT^21uck.

The article "Clinical Features of Acute Coronary Syndrome in Patients with Coronary Heart Disease and Its Correlation with Tumour Necrosis Factor in Cardiology" was published in 2022. Journal: Comput Math Methods Med.

The algorithm iterates until a termination condition is reached, at which point it ceases to operate. The number of points, the linear sum of the points, and the square sum of the points are maintained for each cluster. It is now in the form of a grouping equation,

(14) $$\begin{array}{c} \text{Cluster features}=c\times m\times k^{c}+\zeta . \end{array}$$

Finally, the features can be clustered together and form new signaling feature centroid.

### 3.3. Risk Evaluation

This is the last stage of the process in which the TNF-*α*. After extraction of the features, depending upon the presignaling factor, the level of the production probability of the TNF-*α* can be calculated. It determines the optimal value for each cluster unit,

(15) $$\begin{array}{c} g_{1}\left(s\right)=\frac{\sum_{i\in C_{s}}\left[\overset{⟶}{\text{PBNN}}\left\{GC_{\theta_{q}}\left(q_{i}\right)\right\}⨁\overset{⟵}{\text{PBNN}}\left\{GC_{\theta_{q}}\left(q_{i}\right)\right\}\right]}{\left|C_{s}\right|}. \end{array}$$

All points in the hyperplane fulfil the equation *g*_1_(*s*)=0 that forms the decision boundary between the two classes,

(16) $$\begin{array}{c} Z_{i}g_{i}=\sigma \left({℧}_{z}GC_{\theta_{q}}\left(q_{i}\right)+W_{z}t_{i-1}+b_{g}b_{z}\right). \end{array}$$

Let *Z*_*i*_*g*_*i*_ be the hyper planes which will form a planar area over angle separation,where

(17) $$\begin{array}{c} z_{i}=\sigma \left({℧}_{o}GC_{\theta_{q}}\left(q_{i}\right)+W_{o}t_{i-1}+b_{o}\right),\\ {\hat{Z}}_{i}=\text{tant}\left({℧}_{c}GC_{\theta_{q}}\left(q_{i}\right)+W_{c}t_{i-1}+b_{c}\right). \end{array}$$

The output *c_i_* may be determined by using the sigmoid function, which computes the output of a neuron.

(18) $$\begin{array}{c} c_{i}={g_{i}}^{{}^{\circ}}c_{i-1}+{z_{i}}^{{}^{\circ}}{\hat{c}}_{i}. \end{array}$$

After the feed-forward process is completed, the backpropagation process starts. Let $\overset{⟶}{Y}\;$represent the error-sensitivity and to represent the desired output of a neuron in the output layer. Thus,

(19) $$\begin{array}{c} \overset{⟶}{\;Y}\left(t+1\right)t_{i}=\text{tant}{\left(c_{i}\right)}^{{}^{\circ}}o_{i}. \end{array}$$

After $\overset{⟶}{Y}$ is computed, the weights and biases of each neuron are tuned into backpropagation process by using

(20) $$\begin{array}{c} \underset{U}{\max}\text{imize}\left\{\underset{j}{\sum }\underset{i,i^{\prime }}{\sum }s_{i,i^{\prime },j}U_{i,i^{\prime }}\right\}\text{subject to}\underset{i,i^{\prime }}{\sum }U_{i,i^{\prime }}^{2}\leq 1,\\ \underset{w,U}{\max}\text{imize}\left\{\underset{j}{\sum }w_{j}\underset{i,i^{\prime }}{\sum }s_{i,i^{\prime },j}U_{i,i^{\prime }}\right\}\text{subject to}\underset{i,i^{\prime }}{\sum }U_{i,i^{\prime }}^{2}\leq 1,{\left\|t\right\|}^{2}\leq 1,{\left\|W\right\|}_{1}\\ \leq m,w_{j}\geq 0\forall j. \end{array}$$

As soon as the first input vector has finished fine-tuning the network, the next round of input vectors is ready to be run. Until the network is satisfied with a single output or numerous outputs, the input continues training the networks. Finally depending upon the feature extracted, the TNF_*α* production can be predicted and its severity level can be determined. Depending upon the risk evaluated, it was revealed that the person having the elevated level of the TNF_*α* has the increase risk of coronary syndrome and also those persons have higher risk of getting abnormal hear events in the future due to the elevated upregulated TNF_*α* which was evaluated using the paramount bundle neural network.

The article "Clinical Features of Acute Coronary Syndrome in Patients with Coronary Heart Disease and Its Correlation with Tumour Necrosis Factor in Cardiology" was published in 2022. Journal: Comput Math Methods Med.

## 4. Performance Analysis

In this section, the overall TNF-*α* and lipid levels among study participants were normally evaluated to illustrate their future risk over abnormal coronary events.

Acute coronary syndrome patients were separated into two groups, and their data was collated. Two groups of patients may be shown in Figure 3 with a significant difference in average age and blood pressure. Patients in groups A and B had similar systolic blood pressure readings (58.2 mmHg and 52 mmHg, respectively), as shown by their similar ages.

Figure 4 shows cardiac activity. According to the findings of the research, some people developed heart failure, a myocardial infarction, typical angina, and sudden cardiac death. Heart failure and myocardial infarction were the second and third most prevalent conditions, respectively.

According to the findings, HDL C content was low in both groups A and B before the formation of the coronary syndrome, but it increased considerably following these cardiac events (as shown in Figure 5).

TNF levels were low in both groups before the onset of the cardiac syndrome; however, following the occurrence of the cardiac events, TNF levels increased (Figure 6).

Detection rates for eccentric plaques were compared, as seen in Figure 7. The comparison data indicated that 55.9% and 40.1 percent of the patients in groups A and EB had eccentric plaques.

We can see how different techniques have found different parts of a tumour in Figure 8 (the diameter of the narrowest section). A and B lesions with 2.4 and 2.5 millimetre diameters were revealed to be the two narrowest.

Diastolic blood pressure and thyroglobulin (TG) levels were measured and compared between the two groups (see Figure 9). There were diastolic blood pressure values of 80.38 8.2 mmHg and 84.1 7.8 mmHg, respectively, in groups A and D with TG concentrations of 1.48 and 0.38 mmol/L, respectively. Diastolic blood pressure and serum TG levels were substantially different between the two groups as a consequence (Figure 10).

Prior to the coronary syndrome, group A and group B had CRP levels of 58.5 mmol/L and 59.3 mmol/L, respectively; group B had levels of 70.9 and 78.2. This study found that CRP levels were significantly higher in both groups of patients prior to the onset of coronary syndrome.

The article "Clinical Features of Acute Coronary Syndrome in Patients with Coronary Heart Disease and Its Correlation with Tumour Necrosis Factor in Cardiology" was published in 2022. Journal: Comput Math Methods Med.

Figure 11 shows the comparison results of the detection rate of centripetal plaque. It indicated that the detection rates in group A (48.2%) were obviously lower than those in group B (79.1%).

In Figure 12, you can observe a comparison of LDL-C values in two groups of individuals before and during a coronary syndrome. Before and after the syndrome, LDL-C levels in groups A and B were 2.76 mmol/L and 2.87 mmol/L, respectively; after assessing hormone levels, the probability of cytokine synthesis was predicted using the paramount bundle neural network.

As of from the result obtained from Figure 13, the group B people have the higher risk over abnormal coronary events. From the result obtained, the proposed algorithm can predict the risk level of the patient and their future TNF production rate precisely when compared to other existing mechanisms.

## 5. Conclusions

Patients with an acute coronary syndrome were the focus of this investigation. A control group (group A) and an experimental group (group B) were formed by drawing lots from a hat (group B). These individuals' diagnoses were aided by laboratory testing and a thorough learning evaluation. The accuracy of TNF was compared to traditional methods. For the detection of TNF, a learning algorithm-based prediction technique showed high specificity, accuracy, and sensitivity. Acute coronary syndrome (ACS) may now be clinically identified and treated as a result of the results of this study.

## Figures and Tables

**Figure 1:** TNF-*α* production.

**Figure 2:** Schematic representation of the suggested methodology.

**Figure 3:** Age vs. systolic blood pressure.

**Figure 4:** Cardiac abnormal events.

**Figure 5:** HDL C content evaluation.

**Figure 6:** TNF level evaluation.

**Figure 7:** Detection rate of centripetal plaque.

**Figure 8:** Diameter of narrowest lesion calculation.

**Figure 9:** TG content vs. diastolic blood pressure.

**Figure 10:** CRP content evaluations.

**Figure 11:** Detection rate of eccentric plaque.

**Figure 12:** LDL-C content evaluation.

**Figure 13:** Performance metrics evaluation.

**Algorithm 1:** Paramount bundle neural network.

**Table 1:** Patient characteristics.

	Total number of cases (*n* =272)	Control patients (*n* =272)	Value of *P*
Age in years	50.11 ± 10.80	60.00 ± 9.44	…
Sex	82.90	79.82	…
Smoking status,%	_	_	
Never	20.44	20.72	0.09
Past	54.62	65.91	_
Current	18.61	14.22	_
Level of diabetes	30.11	20.44	0.004
Body metabolic index, kg/m^2^	26.72 ± 5.93	28.55 ± 7.22	0.01
Amount of the blood pressure, mm, hg	_	_	_
Systolic pressure	126.61 ± 18.52	127.90 ± 17.63	0.80
Diastolic pressure	89.11 ± 11.00	79.44 ± 18.62	0.92
Lipid fractions level, mg/dL	_	_	_
Total cholesterol level	209.82 ± 17.81	207.44 ± 18.44	0.44
LDL cholesterol	140.33 ± 14.92	139.33 ± 12.92	0.43
HDL cholesterol	38.22 ± 8.71	39.22 ± 8.55	0.44
Triglycerides	146.55 ± 18.44	149.62 ± 69.55	0.40

The article "Clinical Features of Acute Coronary Syndrome in Patients with Coronary Heart Disease and Its Correlation with Tumour Necrosis Factor in Cardiology" was published in 2022. Journal: Comput Math Methods Med.

## Data Availability

The labeled datasets used to support the findings of this study are available from the corresponding author upon request.
